The article "Rice Plants (Oryza sativa L.) under Cd Stress in Fe Deficiency Conditions" was published in 2022. Journal: Biomed Res Int.

# Rice Plants (*Oryza sativa* L.) under Cd Stress in Fe Deficiency Conditions

**DOI:** 10.1155/2022/7425085

**Published:** 2022-08-08

**Authors:** Saule D. Atabayeva, Agilan B. Rakhymgozhina, Akmaral S. Nurmahanova, Saule S. Kenzhebayeva, Bakdaulet N. Usenbekov, Ravilya A. Alybayeva, Saltanat Sh. Asrandina, Bekzat M. Tynybekov, Aigul K. Amirova

**Affiliations:** Al-Farabi Kazakh National University, Al-Farabi Avenue, 71, Almaty 0050048, Kazakhstan

## Abstract

Due to the environment pollution by cadmium (Cd) near industrial metallurgic factories and the widespread use of phosphorus fertilizers, the problem of toxic Cd effect on plants is well discussed by many authors, but the phytotoxicity of Cd under iron (Fe) deficiency stress has not been sufficiently studied. The aim of the work was to study comprehensively the effect of Cd under Fe deficiency conditions on physiological, biochemical, and anatomical parameters of rice varieties, to identify varietal differences in plant response to the effect of double stress. Relative resistance and sensitivity to the joint effect of Cd and Fe deficiency stress rice varieties have been identified. Double stress decreased a linear growth and biomass accumulation of roots and shoots (by 36-50% and 33-46% and 32-56% and 32-48%, accordingly), content of photosynthetic pigments (Chl*a*, Chl*b*, and carotenoids by 36-51%, 32-47%, and 64-78%, accordingly), and relative water content (by 18-26%). Proline content increased by 28-103% in all rice varieties, but to a lesser extent in sensitive varieties. The thickness of the lower and upper epidermis and the diameter of vascular bundles of leaves decreased by 18-50%, 46-60%, and 13-48%, accordingly. The thickness of the root endodermis and exodermis and diameter of the central cylinder mainly decreased. The thickness of the exodermis increased slightly by 7%, and the diameter of the central cylinder remained at the control level in resistant Madina variety while in sensitive Chapsari variety, these indicators decreased significantly by 50 and 45%, accordingly. Thus, the aggravation of adverse effect of Cd under Fe deficiency conditions and the varietal specificity of plants' response to double stress were shown. It creates the need for further study of these rice varieties using Fe to identify mechanisms for reducing the toxic effect of Cd on plants as well as the study of Fe and Cd transporter genes at the molecular level.

## 1. Introduction

Environmental pollution with heavy metals has a toxic effect on human health, as they can accumulate in the body. The high rate of industrialization entails an increase in heavy metal pollution around industrial enterprises in many countries [1]. The wastes of many industries contain heavy metals in their composition. Among heavy metals, cadmium (Cd) is highly toxic to living organisms even at low amounts. According to the International Agency for Research on Cancer (IARC), Cd is a strong carcinogen for humans. Human exposure to Cd mainly occurs when consuming contaminated food products and when inhaling polluted air by employees of metallurgical enterprises [2, 3].

The article "Rice Plants (Oryza sativa L.) under Cd Stress in Fe Deficiency Conditions" was published in 2022. Journal: Biomed Res Int.

In Kazakhstan, rice is an important import-substituting and export crop. The total area of the engineered systems for rice cultivation is about 225000 ha [4]. Therefore, to ensure food security, the development of rice farming in Kazakhstan is an important strategic task [5].

Heavy metal pollution is a big problem, as heavy metals around metallurgical factories, as well as around mining deposits, accumulate in large amounts in the soil and are transmitted along the food chain [6, 7]. Cd is usually present in trace amounts in the soil. The functioning of metallurgical enterprises and the use of phosphogypsum on saline soils, which contains Cd in its composition, also contribute to its accumulation [8, 9]. Cd is found in the composition of phosphorite rocks, which are used in the production of phosphorus fertilizers [10, 11]. The widespread application of phosphorus fertilizers increases the accumulation of Cd in the soil [12–17]. Cd is a very mobile element and easily moves through the phloem to other parts of plants [18, 19]. When Cd ions enter the human body, it causes various diseases [20, 21]. Rice grown on contaminated soils, especially in Southeast Asia, as well as in other contaminated regions, is the main source of Cd intake in the human body along with food [22]. Cd, which has high mobility in the soil, enters plants through the roots and moves through all parts of plants and causes multiple symptoms of toxicity [23]. The level of Cd accumulation in plants depends on many factors, such as its total content in the soil, biological availability, genetic features of plants, soil properties, and the rhizosphere [24–26]. Cd negatively affects the growth and development of plants, and it has a negative impact on various physiological and biochemical processes, but plants have developed various resistance mechanisms to reduce Cd toxicity [27]. Under Cd stress, growth parameters decrease and physiological and biochemical processes are disrupted—the content of photosynthetic pigments and the intensity of photosynthesis decrease, and water absorption, mineral nutrition, and carbohydrate metabolism are disrupted [28–30].

The decline of plant biomass is a result of the alterations in the photosynthesis process. It was found that Cd affects stomatal conductivity, and its index is affected by transpiration and the net rate of photosynthesis [31]. It was revealed that Cd reduced the photochemical efficiency of PSII. It is assumed that a strong decrease in plant growth is a consequence of a decrease in the absorption of CO_2_, which occurs due to a decline in the activity of the enzyme Rubisco. Also, under Cd stress, the absorption of nutrients and carbohydrates decreases [32]. It was found that under heavy metal stress, the carbohydrate content decreases due to violation of biosynthesis of chlorophyll. The greatest reduction in carbohydrate content was shown with Cd stress compared to exposure to lead (Pb) and copper (Cu) [33]. Oxidative stress caused by Cd disrupts important biochemical and physiological processes in plants, which have a negative impact on growth and metabolic processes and accelerate aging [34, 35]. Reactive oxygen species (ROS) can damage proteins, nucleic acids, and amino acids and cause lipid peroxidation [36–39]. It was revealed that Cd reduces the content of the main macro- and microelements in plants [40–42]. There is an antagonistic interaction in plants between Cd and mineral elements such as Fe, manganese (Mn), Cu, and Zn [27].

The article "Rice Plants (Oryza sativa L.) under Cd Stress in Fe Deficiency Conditions" was published in 2022. Journal: Biomed Res Int.

There are chemical similarities between divalent cations like Zn^2+^, Fe^2+^, Ca^2+^, and Cd^2+^. Cd ions can be transported by transporters of Ca^2+^ and Zn^2+^[43]. The excess of Cd in the soil reduces the assimilation of important nutrients by plants, such as Zn, Mn, and Fe, due to their competition on the surface of the roots. The appearance of chlorosis and necrosis of leaves and a decrease in plant height are physical symptoms of Cd toxicity [44]. Rolling of leaves, closure of stomata, and reduced water content are the symptoms of Cd toxicity in plants. It is assumed that changes in the ratio Fe/Zn and the negative influence of Cd on the metabolism of chlorophyll are the causes of leaf chlorosis under Cd stress [45]. Mineral elements like as Fe, sulfur (S), and silicon (Si) reduce Cd poisoning to higher plants, preventing its accumulation [46].

Fe is the most effective and potentially important trace element among minerals, which plays a key role in reducing the toxicity of heavy metals. It has been established that the use of Fe to decrease the toxic effects of metals on plants is effective. It was found that Fe absorption reduces Cd intake in plants, while Fe deficiency enhances Cd accumulation in plants [47–49]. On the contrary, the deficiency of Fe leads to increased absorption and accumulation of Cd [50, 51]. It was shown that Cd (5, 20, and 40 *μ*M) decreases Fe content in the leaves and roots of *Arabidopsis thaliana*. Cd (40 *μ*M) reduced the content of elements such as Zn, Mn, and calcium (Ca) [52]. It was found that Cd reduces the rate of Fe transport from roots to the aboveground parts in *Brassica napus*, and a rapid increase in the Fe content in the roots and the Fe deficiency in the aboveground organs were also detected [53]. The Fe content in xylem and phloem considerably decreased, while content of Cd increased [54]. It was determined that the differential sensitivity of some transporter genes to Fe deficiency is associated with high or low Cd accumulation in *Solanum* species [55]. Cd absorption is carried out by transporters such as the family of Zn- and Fe-regulated transporters (ZIP), heavy metal-transporting ATP-ases (HMA), and the family of natural resistance-associated macrophage proteins (NRAMP) that participate in the intake of basic mineral elements. They can also transport divalent metal ions (Cd^2+^, Fe^2+^, Cu^2+^, Ni^2+^, Mn^2+^, Zn^2+^, and Co^2+^) [1, 56–59]. It has been shown that Fe transporters OsIRT1 and OsIRT2 and Zn transporter OsZIP1 can also serve as Cd transporters [60].

The article "Rice Plants (Oryza sativa L.) under Cd Stress in Fe Deficiency Conditions" was published in 2022. Journal: Biomed Res Int.

NRAMP consists of a conservative family of integral cell membrane proteins that are involved in the transport of Fe [1, 61]. Fe transporters such as OsNRAMP1 and OsNRAMP5 are also considered Cd transporters in the plasma membrane [62]. AtNRAMP6 belongs to Cd transporters inside the cell [63]. The content of Fe in the soil is usually high, but iron is mainly in insoluble form (Fe^3+^), particularly in aerobic conditions and at high pH. This is the reason for the lack of available forms of Fe [64, 65]. Since plants usually absorb Fe from the soil in the form of Fe^2+^, a deficiency of available Fe in the soil leads to Fe deficiency in plants [66]. Fe is essential in plant metabolism; it is a component of the electron transport chain in the processes of photosynthesis, respiration, and fixation of molecular nitrogen [67–70]. Fe is necessary for the synthesis of specific chlorophyll protein complexes in chloroplasts, and under Fe deficiency conditions, yellowing of leaves is observed and photosynthetic activity decreases [71]. Fe also is a cofactor for some enzymes [72]. Fe deficiency reduces the content of Fe-containing components in chloroplasts, such as Fad (ferredoxin protein Fe-S) [73].

Fe deficiency in soils can be observed at very high and at very low pH [74]. It was found that Cd in the nutrient medium exacerbates Fe deficiency. Leaf chlorosis, similar to chlorosis due to Fe deficiency, is one of the visual signs of Cd toxicity. Some studies have shown that under Cd stress, a translocation of Fe from the roots to the aboveground organs decreased, which contributes to a decrease in the synthesis of chlorophyll in plant leaves [27, 75–77]. For Cd accumulation by plants, the process of its absorption by plant roots is the key point. In radish plants, Cd significantly reduced the accumulation of biomass, increased the content of malondialdehyde and increased the permeability of membranes, and reduced the content of chlorophyll and the absorption of mineral nutrients such as Fe, K, and Ca. After application of Fe-enriched biochar (Fe-BC), Cd toxicity to plants was reduced, the activity of antioxidant enzymes such as heme-based ascorbate peroxidase (APX) was enhanced, the accumulation of primary and secondary metabolites increased, and the mineral nutrition of plants improved. It is assumed that Fe-BC regulates the activity of the peroxidase enzyme and supports redox homeostasis [78]. It has also been established that Fe activates the APX1 gene and regulates the expression of the activity of the cytosolic enzyme APX [79, 80]. It has been revealed that genes associated with the absorption and transport of Fe can play a crucial role in reducing Cd accumulation and increasing plant resistance to it. It follows that uptake, transport, and accumulation of Cd in grains of rice can be lowered by creating genotypes that limit Cd uptake. To do this, CRISPR/Cas9 technologies can be used for knocking out or editing these genes [81]. Cd loading into the xylem and its translocation with other plant organs can be controlled by the expression of the OsHMA2 gene [82], and the expression of OsNRAMP5 and OsLCT1 is associated with Cd phloem transport [62]. To identify new genes is needed to better understand Cd transport and its accumulation in rice plants [83].

The article "Rice Plants (Oryza sativa L.) under Cd Stress in Fe Deficiency Conditions" was published in 2022. Journal: Biomed Res Int.

It was revealed that the adsorption of Cd by oxides of Fe(III) increased with an increase in pH to 6.5, which reduces the content of dissolved Cd in the soil [84]. It has been shown that the Fe plaque persists at a pH level above 6.5 and disappears at a pH level below 4.5 [85]. Due to continuous flooding and weekly alternation of humidification and drying in naturally polluted rice soil, a pH of 4.29-8.62 is achieved. This contributes to the transformation of crystal Fe (III) oxide into a formless state, which leads to better immobilization of Cd and significantly reduces the availability of Cd in the soil [86–88].

Also, it was shown that Fe nanoparticles (Fe NPs) are specific strong adsorbents that have an original structure and electronic features. Magnetic Fe nanoparticles can be separated from the absorbent medium using a magnetic field [69]. The mechanism of operation of nano-Fe is that it adsorbs heavy metals, stimulates the formation of a Fe film on the surface of the root, and activates the antioxidant system [89]. It is assumed that Fe-Si-Ca, organic fertilizers, and biocoal from coconut shells contributed to an increase in the cadmium phytostabilizing ability of *Boehmeria nivea* L. plants [90, 91]. Nano-Fe and Fe-containing fertilizers can be used for increasing plant growth [92]. It was shown that nanoscale zero-valent Fe (nZVI) reduced the accumulation of heavy metals in sunflowers, increased superoxide dismutase (SOD) and peroxidase (POD) activities in plant leaves, and promoted plant growth [92].

The article "Rice Plants (Oryza sativa L.) under Cd Stress in Fe Deficiency Conditions" was published in 2022. Journal: Biomed Res Int.

It was demonstrated that after application of nZVI to rice seedlings, expression of genes of YSL2, YSL15, IRT1, and IRT2 that are responsible for Cd and Fe uptake was downregulated. On the contrary, overexpression of OsVIT1 and OsCAX4 genes leads to isolation of Cd in vacuoles [93]. It was shown that soil and foliar application of Fe_2_O_3_-NPs (5-20 ppm) under Cd stress reduced Cd content in grains, the dry weight, and the electrolyte leakage of leaves and enhanced the activity of antioxidant enzymes of wheat [94]. It was demonstrated that the foliar application of Fe-NPs is more preferable. Foliar application of Fe NPs has mitigating effects on Cd stress in rice, and this effect was enhanced by application of biochar [95]. But in other study, biochar-Fe_3_O_4_ nanocomposites contributed to greater Cd mobility in water-saturated soil, which indicates that not all risks have been studied yet [96].

It was shown that drought aggravated the negative effect of Cd on plants. The addition in the soil of Fe_2_O_3_ NPS improved photosynthesis indicators, increased productivity, and decreased the content of Cd in grain of wheat [97]. Spraying of these Fe materials has been shown to reduce DNA damage caused by Cd, and the positive effect of NPS Fe_2_O_3_ was more pronounced than that of FeCl_3_. Also, the effect of foliar application of Fe_2_O_3_-NPs and FeCl_3_ for seedlings rice plants was studied (Hybrid Rice Y Liangyou 900), growing hydroponically with 50 *μ*M CdCl_2_[98]. It was shown that spraying of these Fe materials reduces damage of DNA, caused by Cd, and the positive effect of NPS Fe_2_O_3_ was more pronounced than that of FeCl_3_.

The results of these studies on the use of Fe compounds in organic fertilizers and foliar application of iron nanoparticles indicate a significant role of Fe to reduce Cd phytotoxicity. The Fe deficiency in the growth medium under Сd stress is a significant factor, influencing the toxicity of Cd for plants. But the impact of Fe deficiency on the phytotoxicity of Cd at physiological, biochemical, and anatomical parameters under Cd stress and the varietal specificity of this effect have not been sufficiently studied. Based on the above, the objective of our work was to study comprehensively the joint effect of Cd and Fe deficiency on rice varieties, identify resistant rice varieties to separate and joint effects of these stress factors, and reveal the degree of the effect of different Fe status in nutrient medium on the phytotoxicity of Cd.

The article "Rice Plants (Oryza sativa L.) under Cd Stress in Fe Deficiency Conditions" was published in 2022. Journal: Biomed Res Int.

## 2. Materials and Methods

Rice plants (*Oryza sativa* L.) of 4 varieties Madina, Bakanas, Barakat, and Chapsari were grown under hydroponic conditions in plastic containers in 3 replicates each variant (3 × 4 variants = 12). Plants were grown 14 days in a nutrient medium containing the main mineral elements in factor static conditions at 22°C during the day and 18°C at night, with a 14-hour photoperiod, at light intensity of 61 *μ*mol m^−2^ s^−1^. The variants differed in the content of Fe and Cd in the nutrient solution (nutrient medium content: K_2_SO_4_—0.70 mM, KCl—0.10 mM, KH_2_PO_4_—0.10 mM, Ca(NO_3_)_2_—2.0 mM, MgSO_4_—0.50 mM, H_3_BO_3_—10 *μ*M, MnSO_4_—0.50 *μ*M, CuSO_4_—0.20 *μ*M, (NH_4_)_6_Mo_7_O_24_—0.01 *μ*M, and ZnSO_4_—0.5 *μ*M), and Fe in concentration 100 *μ*М was added as Fe(III)-EDTA (pH 6.0) [99]. Rice plants were grown up to 14 days in the following variants: (1) control-Fe norm-Cd (nutrient medium (NM)+100 *μ*М Fe), (2) Fe norm+Cd (NM+100 *μ*М Fe+200 *μ*М Сd), (3) Fe deficiency-Cd (NM+0 *μ*М Fe), and (4) Fe deficiency+Cd (NM+0 *μ*М Fe +200 *μ*М Сd). The measurement of growth parameters was carried out as follows: the plants were separated into aboveground organs and roots, and the length of roots and aboveground organs was measured. To determine the dry biomass, the plants were placed in a dry-burning cabinet and dried at 105°C to a constant weight, cooled to room temperature, and weighed.

Photosynthetic pigments were determined by spectrophotometry. Extraction of chlorophyll and carotenoid was carried out by using acetone [100]. Samples of plant material (0.3-0.5 g) were ground in a porcelain mortar with a small amount of 80% acetone (2-3 ml) and pure quartz sand; then, it was filtered. The supernatant was transferred, and the procedure was repeated till the residue becomes colourless. Then, they were infused (2-3 minutes) with subsequent filtration. The resulting extract was filtered through a filter paper from a funnel into flasks of 25 ml and passed for 10 ml. The chlorophyll pigments and carotenoid concentrations were determined based on the absorbance of three wavelengths: 649, 665, and 440.5 nm. Concentrations of chlorophyll pigments were calculated according to the equation of Vernon [101]:

(1) $$\begin{array}{c} \begin{array}{c} \text{Ca}\left(\text{mg}/\text{L}\right)=11.63\times \text{D}665-2.39\times \text{D}649\\ \text{Cb}\left(\text{mg}/\text{L}\right)=20.11\times \text{D}649-5.18\times \text{D}665 \end{array}, \end{array}$$

The carotenoid content was determined by Von Wettstein's equation [102]:

(2) $$\begin{array}{c} \text{Ccar }\left(\text{mg}/\text{L}\right)=4.695\times \text{D}440.5-0.268\times \left(\text{Ca}+\text{Cb}\right). \end{array}$$

Content of photosynthetic pigments was calculated according the following equation:

(3) $$\begin{array}{c} A=\frac{C\times V}{P\times 1000}, \end{array}$$

where *A* is the content of pigments (mg/g); Ca and Cb are concentrations of chlorophylls *a* and *b* (mg/l); Ccar is the concentration of carotenoids (mg/l); D665, D649, and D440.5 are optical densities of solutions at corresponding wavelengths; *V* is the volume of the extractant (ml); and *P* is the weight of the plant leaf sample (g).

(4) $$\begin{array}{c} A=\frac{C\times V}{P\times 1000}, \end{array}$$

where *A* is the content of photosynthetic pigments (mg/g, wet weight), *C* is the concentration of photosynthetic pigments (mg/l), *V* is the volume of the extractant (ml), and *P* is the weight of the leaf sample (g).

The article "Rice Plants (Oryza sativa L.) under Cd Stress in Fe Deficiency Conditions" was published in 2022. Journal: Biomed Res Int.

The proline content is determined by Bates et al. with ninhydrin [103].

A sample of fresh plant leaves (200 mg) was poured with 5-20 ml boiling distilled water and kept for 30 minutes in a water bath at a temperature of 100°C. Then, 1 ml of glacial acetic acid and 1 ml of ninhydrin reagent were poured into a clean test tube, and 1 ml of the prepared extract was added. The samples were incubated for 60 minutes in a water bath, after which it was quickly cooled to room temperature. After cooling (with cold water or ice), the optical density was determined on a spectrophotometer at a wavelength of 520 nm. The concentration of proline was determined using a calibration curve. The calculation of proline content was performed by the following formula:

(5) $$\begin{array}{c} A=\frac{nV}{P}, \end{array}$$

where *A* is the proline content, *n* is the value according to the calibration curve, *V* is the dilution volume (ml), and *P* is the weight of the sample (g).

The relative water content (RWC) in the leaves was determined using the method described by Schonfeld et al. [104]. It is necessary to determine the fresh weight (FW), turgor weight (TW), and dry weight (DW) of plant leaves. Five seedlings were taken from each variant, and the raw mass of the plant (FW) was measured. After that, the leaves were incubated with distilled water for 16-18 hours. The turgor weight (TW) of the plant was determined after incubation. Before the measurement, the samples were dried with filter paper to get rid of excess moisture. The samples were dried for 72 hours at 70°C. After drying, the dry weight (DW) of the plant sample was determined. After all the measurements were obtained, the relative amount of water (RWC) was determined using the following equation:

(6) $$\begin{array}{c} \text{RWC}=\left(\frac{\text{FW}–\text{DW}}{\text{TW}-\text{DW}}\right)\times 100, \end{array}$$

where RWC is the relative water content (%), FW is the raw weight of the plant sample (g), TW is the turgor weight (g), and DW is the dry weight of the plant sample (g).

The article "Rice Plants (Oryza sativa L.) under Cd Stress in Fe Deficiency Conditions" was published in 2022. Journal: Biomed Res Int.

Microscopic studies were carried out on the plant material. It was fixed in a mixture, containing alcohol, glycerin, and water (1 : 1 : 1). For anatomical studies, generally accepted methods in plant anatomy were used [105–107]. Anatomical specimens were made by a microtome with a freezing device OL-ZSO (InMedProm, Russia), with a double concave blade. The anatomical sections have a thickness 10-15 microns. For quantitative analysis, morphometric parameters were measured with an ocular micrometer MOV-1-15 (by a lens ×9, magnification ×10.7). Micrographs of anatomical sections were taken on a microscope MC300 (Micros, Austria) with a video camera CAMV400/1.3M (JProbe, Japan).

Statistical data processing was carried out using two-way analysis of variance with varieties and treatments as the main factors and one-way variance analysis to determine the significance of the difference between control and treatments using the Statistica 11.5 package and Excel 2010 from the Microsoft Office XP package. In the figures, the values are marked with asterisks for the significance level as compared to the control. All values were expressed as the average of 3 measurements for each treatment. The number of replications is 3, and each measurement was conducted using plant seedlings from 3 separate growth plastic containers for each variant. Values were represented as means ± standard error (SE).

## 3. Results and Discussion

### 3.1. The Effect of Cd and Fe Deficiency on the Growth Parameters of Rice Seedlings

The separate and joint effect of Cd and Fe deficiency stress on growth parameters of rice seedlings was negative (Figures 1 and 2). Cd and Fe deficiency caused inhibition of growth of aboveground organs as well as roots. The length of rice plant shoots of 14 d rice seedlings decreased in the following order (% to control): Fe norm+Cd—Madina (86) > Bakanas (77) > Barakat (72) > Chapsari (63); Fe deficiency-Cd—Madina (89) > Bakanas (86) > Barakat (83) > Chapsari (70); and Fe deficiency+Cd—Madina (68) > Bakanas (66) > Barakat (59) > Chapsari (44).

Cadmium stress and Fe deficiency decreased the biomass of the shoots of 14 d seedlings of rice plants. The degree of reduction in the biomass of aboveground rice organs in variants with different Fe and Cd contents increased in the following order (% to control): Fe norm+Cd—Madina (77) > Bakanas (74) > Barakat (63) > Chapsari (61); Fe deficiency-Cd— Madina (88) > Bakanas (83) > Barakat (78) > Chapsari (76); and Fe deficiency+Cd—Madina (68) > Bakanas (63) > Barakat (57) > Chapsari (52).

The article "Rice Plants (Oryza sativa L.) under Cd Stress in Fe Deficiency Conditions" was published in 2022. Journal: Biomed Res Int.

The biomass of the shoots in Madina, Bakanas, Barakat, and Chapsari varieties in different variants decreased in the following order (% to control): Fe deficiency‐Cd (88, 83, 78, and 76) > Fe norm + Cd (77, 74, 63, and 61) > Fe deficiency + Cd (68, 63, 57, and 52).

In the presence of Fe under Cd stress, the biomass of aboveground organs decreased in rice varieties to various degrees (Figure 1). It was observed that the dry weight of the shoots of 14 d seedlings of rice varieties decreased by 23, 26, 37, and 39% in the varieties Madina, Bakanas, Barakat, and Chapsari, respectively, and the biomass of Barakat and Chapsari varieties decreased to the greatest extent.

The Fe deficiency also reduced the accumulation of biomass in the aboveground organs of rice seedlings. Chapsari plants suffered the most from the Fe deficiency (by 24%).

But double stress, both Fe deficiency and the effect of Cd, significantly reduced the biomass accumulation in shoots of rice seedlings. In all the studied varieties, the greatest decrease in biomass relative to the control variant was observed in variant “Fe deficiency+Cd” by 32, 37, 43, and 48% in Madina, Bakanas, Barakat, and Chapsari varieties, respectively. The most affected varieties were Barakat and Chapsari.

Root growth also decreased under the effect of Fe deficiency and excess of Cd with joint and separate effect. The reduction in the root length of 14 d rice seedlings can be reflected in the following order (% to control) (Figure 3 and 4): Fe norm+Cd—Madina (83) > Bakanas (77) > Barakat (71) > Chapsari (66); Fe deficiency-Cd— Madina (87) > Bakanas (82) ≥ Barakat (82) > Chapsari (79); and Fe deficiency+Cd—Madina (64) > Bakanas (61) ≥ Barakat (58) > Chapsari (50).

The level of the root length decrease in Madina, Bakanas, Barakat, and Chapsari varieties can be presented in the following order (% to control): Fe deficiency‐Cd (87, 83, 82, and 79) > Fe norm + Cd (82, 77, 71, and 66) > Fe deficiency + Cd (64, 61, 58, and 50).

The root dry weight also decreased to varying degrees in different varieties of rice (% to control) (Figure 3): Fe norm+Cd—Madina (73) > Bakanas (68) = Barakat (68) ≥ Chapsari (67); Fe deficiency-Cd— Bakanas (88) > Madina (84) > Barakat (79) ≥ Chapsari (78); and Fe deficiency+Cd—Bakanas (67) > Madina (66) > Barakat (59) > Chapsari (54).

The article "Rice Plants (Oryza sativa L.) under Cd Stress in Fe Deficiency Conditions" was published in 2022. Journal: Biomed Res Int.

The variants by the level of decrease for Madina, Bakanas, Barakat, and Chapsari varieties are shown in the following order (% to control): Fe deficiency‐Cd (88, 84, 79, and 78) > Fe norm + Cd (73, 68, 68, and 67) > Fe deficiency + Cd (67, 66, 59, and 54).

The decrease in linear growth and biomass accumulation by rice seedlings was observed under Fe deficiency conditions. Fe deficiency aggravated the inhibitory effect of Cd on rice plant growth in our studies. The greatest decrease in the growth parameters of roots and aboveground organs was observed in the variant with Fe deficiency under Cd stress. The same results have been shown by other researchers.

According to other researchers, it is known that Fe deficiency reduces plant productivity [108], protein synthesis in leaf chloroplasts [109], the activity of Rubisco (ribulose-1,5-bisphosphate carboxylase/oxygenase) activity [110], the activity of photosystem 2 (PSII), and the content of photosynthetic pigments [111]. It was found that the rate of photosynthesis measured before flowering is a good indicator of productivity for grain sorghum. There is a correlation between the rate of photosynthesis and productivity of plants. Therefore, violations of photosynthesis processes entail negative phenomena such as a decrease in growth parameters and a decrease in biomass accumulation [112, 113]. The results of many studies show that Cd reduces the productivity of plants, inhibits their development, and disrupts photosynthesis, water balance, ion exchange, and mineral nutrition, which leads to inhibition of linear growth and accumulation of biomass by plants [53, 114, 115].

The supply of important nutrients in the required amounts is necessary for better plant growth, because they create the structure and functional components of the cells. It has been established that an excess of Cd in the growing medium disrupts the mineral nutrition of plants. There is a negative correlation between the absorption and distribution of the necessary macro- and microelements in various plant organs under Cd stress [41, 53, 116]. The first target of the negative effect of Cd is the cell membrane, as well as transporters that participate in the absorption of K, Mn, and Mg elements [117]. It was found that Cd absorbed by plant roots enters the cell through the plasmalemma using the ZIP family of transporters (ZRT-IRT-like protein, Zn-regulated transporter, and Fe-regulated transporter) and NRAMP. Cd competes with the main nutrients [50, 60], is transferred to the aboveground organs, and leads to a decrease in growth. A decrease in growth rates and yields with an increased Cd content in nutrient media leads to leaf rolling and leaf and stem chlorosis [29] and reduces gas exchange [118]. The negative effect of Cd on the absorption of mineral elements is explained by a decrease in transpiration due to a decrease in the conductivity of stomata [119], and the consequence of a decrease in root growth is a decrease in their absorption of mineral elements from the soil [120].

The article "Rice Plants (Oryza sativa L.) under Cd Stress in Fe Deficiency Conditions" was published in 2022. Journal: Biomed Res Int.

Photosynthesis is a fundamental, well-organized, and consistent process involving photosynthetic pigments and photosystems, an electron transport system, and ways of assimilation of CO_2_. Multiple damage caused by Cd, at any level, has a negative effect on photosynthesis in general [121]. A decrease in the photochemical efficiency of PSII was observed under Cd stress (at 10 and 50 *μ*M). The decrease in CO_2_ assimilation due to the decrease in Rubisco activity led to a strong inhibition of plant growth in the presence of Cd in growing medium. Cd also changes the nutrition of various parts of plants, which can also have great physiological significance for photosynthesis [29, 122, 123]. Electron transport in PSI and PSII photosystems is also disrupted; the Kelvin cycle was disrupted, reducing Rubisco activity under Cd stress [124, 125]. Cd caused the stomata closure due to its entry into the guard cells of the stomata instead of Ca^2+^[126], and the content of stomata per unit area decreased [127]. It has been shown that Cd affects the conductivity of stomata, and its index is influenced by transpiration and the net rate of photosynthesis [128]. Cd stress reduced the net photosynthesis rate in *Brassica juncea* L. varieties, which corresponded to a decrease in the activity of Rubisco and carbonic anhydrase (CA) [129]. Under the influence of Cd, a decrease in the amount of chlorophylls (Chl(*a*+*b*), Chl*a*, and Chl*b*) was observed to varying degrees in *Brassica juncea* L. varieties [129], which may be a consequence of violated chlorophyll biosynthesis [123].

Thus, the decrease in growth parameters of rice seedlings, like length and biomass accumulation of vegetative parts, was observed. According to data of other researchers, there is a result of changes in biochemical and physiological processes under Cd stress in Fe deficiency conditions, in particular, decrease in photosynthetic rate and content of photosynthetic pigments. Therefore, the next step was the study of the Cd effect on chlorophyll and carotenoid content in different Fe status in rice plants.

### 3.2. The Effect of Cd and Fe Deficiency on the Content of Photosynthetic Pigments in the Leaves of Rice Seedlings

The effect of Cd and Fe deficiency on the content of chlorophyll *a* in the leaves of 14-day rice seedlings was evaluated. In all variants, the content of chlorophyll *a* (Chl*a*) decreased relative to the control in all the studied rice varieties. The degree of reduction in the content of Chl*a* in rice seedlings of Madina, Bakanas, Barakat, and Chapsari varieties was determined; the following pattern was observed (% to control, respectively): Fe deficiency‐Cd (86, 82, 80, and 73) > Fe norm + Cd (70, 71, 60, and 56) > Fe deficiency + Cd (64, 61, 53, and 49) (Figure 5).

The article "Rice Plants (Oryza sativa L.) under Cd Stress in Fe Deficiency Conditions" was published in 2022. Journal: Biomed Res Int.

In all the studied varieties, the greatest decrease in Chl*a* content was observed in variant “Fe deficiency+Cd” by 36, 39, 47, and 51% in varieties Madina, Bakanas, Barakat, and Chapsari, respectively.

The greatest decrease in this variant was found in the Chapsari variety (% to control): Fe norm+Cd— Bakanas (71) ≥ Madina (70) > Barakat (60) > Chapsari (56); Fe deficiency-Cd— Madina (86) > Bakanas (82) > Barakat (80) > Chapsari (73); Fe deficiency+Cd—Madina (64) > Bakanas (61) > Barakat (53) > Chapsari (49).

Content of Chl*b* was decreased in the following order (% to control) (Figure 6): Fe norm+Cd—Madina (80) > Bakanas (72) > Chapsari (71) ≥ Barakat (65); Fe deficiency-Cd—Madina (89) > Bakanas (86) > Barakat (84) > Chapsari (80); and Fe deficiency+Cd—Madina (68) ≥ Bakanas (60) > Chapsari (54) ≥ Barakat (53).

The following degree of reduction in the content of Chl*b* in Madina, Bakanas, Barakat, and Chapsari varieties was observed (% to control, accordingly): Fe deficiency‐Cd (89, 86, 84, and 80) > Fe norm + Cd (80, 72, 71, and 65) > Fe deficiency + Cd (60, 50, 53, and 54).

In all the studied varieties, the greatest decrease in the content of Chl*b* relative to the control was observed in variant “Fe deficiency+Cd” by 20, 28, 29, and 35% in varieties Madina, Bakanas, Barakat, and Chapsari, respectively. The greatest decrease in this variant was found for the Chapsari variety.

### 3.3. The Effect of Cd and Fe Deficiency on the Content of Carotenoids in the Leaves of Rice Seedlings

The following pattern was observed in carotenoid content in rice varieties (% to control) (Figure 7): for Madina variety— Fe norm + Cd (93) > Fe deficiency‐Cd (54) > Fe deficiency + Cd (36); for Bakanas variety— Fe norm + Cd (120) > Fe deficiency‐Cd (83) > Fe deficiency + Cd (25%); for Barakat variety— Fe norm + Cd (100) > Fe deficiency‐Cd (62) > Fe deficiency + Cd (41); and for Chapsari variety— Fe norm + Cd (71) > Fe deficiency‐Cd (41) > Fe deficiency + Cd (22).

In different variants, carotenoid content can be presented in the following order (% to control): Fe norm+Cd— Bakanas (105) ≥ Madina (93) > Barakat (100) > Chapsari (71); Fe deficiency-Cd— Bakanas (83) > Madina (54) > Barakat (62) > Chapsari (41); and Fe deficiency+Cd—Madina (36) = Bakanas (25) > Barakat (15) > Chapsari (22).

The article "Rice Plants (Oryza sativa L.) under Cd Stress in Fe Deficiency Conditions" was published in 2022. Journal: Biomed Res Int.

It was found that in variant “Fe norm+Cd” in Madina, Bakanas, and Barakat cvs, carotenoid content slightly changed or did not change, while in Fe deficiency condition and under double stress in variant “Fe deficiency+Cd” in all rice varieties, carotenoid content decreased.

The most decline of carotenoid content was observed in Chapsari cv.

Thus, chlorophyll and carotenoid content in leaves of rice seedlings decreased under Cd stress and in most degrees under joint effect of Cd stress and Fe deficiency conditions.

The data obtained are consistent with the results of studies by other authors. According to other studies, plant photosynthetic systems are specific targets of Cd [130]. According to the researchers, photosynthetic systems are severely damaged by an increase in the level of Cd in the growing medium, a decrease in the content of chlorophyll, and the assimilation of carbon by the enzyme Rubisco. It has been found that Cd inhibits chlorophyll biosynthesis, increases its breakdown, disrupts carboxylation reactions as well as photochemical reactions of photosynthesis, and generally destroys chloroplast metabolism [131]. Leaf chlorosis as a result of Cd toxicity was directly associated with a decrease in the level of chlorophyll biosynthesis in rice plants [116] as well as mungbean [29], peas [40], and brassica [122].

High concentrations of Cd prevent the incorporation of Mg^2+^ into protoporphyrinogen and cause the breakdown of chlorophylls (Chl*a* and Chl*b*) [121].

It is assumed that the decrease in the content of chlorophyll may be associated with increased activity of chlorophyllase, which destroys chlorophylls, or with a decrease in the activity of a crucial enzyme in the biosynthesis of chlorophyll, 5-aminolevulinic acid dehydratase (ALAD) [132]. It was established that in Fe deficiency conditions caused by Cd, the development of thylakoid membranes and the synthesis of chlorophylls and chlorophyll-protein complexes are disrupted, as a result of which the composition of the thylakoid is modified [133].

Fe deficiency causes destructions in the structure and functions of the entire photosynthetic apparatus in higher plants. The reduction in pigment content caused by Fe deficiency seems to be related to the absolute need for Fe in the formation of the thylakoid membrane.

Under conditions of iron deficiency in leaf thylakoids, disturbances were observed in the stoichiometry of PSII and PSI, in the ratios of chlorophylls and xanthophylls, and in their lipid profile [134].

It can be noted that in the Bakanas variety, carotenoid content slightly increased (by 5%), and in Barakat cv, it did not change. Content of carotenoids increases [135, 136] or decreases [51, 137] under Cd stress in different studies.

The article "Rice Plants (Oryza sativa L.) under Cd Stress in Fe Deficiency Conditions" was published in 2022. Journal: Biomed Res Int.

Carotenoids are low-molecular-weight antioxidants [138], so an increase in their amount under stressful conditions indicates the activation of protective functions. Maintenance of a stable level of pigments of photosynthesis is an important demonstration of plant resistance to heavy metals [132]. Besides their photochemical function, carotenoids significantly alleviate the oxidative damage in membrane thylakoids caused by adverse environmental conditions [139]. In our studies in Fe-deficient conditions, chlorophyll content and carotenoid content decreased in all varieties. Other researches obtained the same results. It was established that Fe deficiency causes a reduction of chlorophyll and carotenoid content [140, 141]. Joint effect of Cd and Fe deficiency stress amplified the negative separate effect of these stresses.

### 3.4. The Effect of Cd at Different Fe Status on the Relative Water Content (RWC) in the Leaves of Rice Seedlings

Unfavorable conditions for plant growth cause a decrease in water content in plant parts [69, 87]. Relative water content in leaves of rice seedlings, subjected to Cd and Fe deficiency stresses and their joint effect, was studied.

Relative water content (RWC) in different rice varieties decreased in the following order (% to control) (Figure 8): Fe norm+Cd—Madina (92) > Bakanas (90) > Chapsari (84) = Barakat (84); Fe deficiency-Cd— Madina (93) ≥ Bakanas (92) = Barakat (86) > Chapsari (83); and Fe deficiency+Cd—Madina (82) > Bakanas (79) > Barakat (75) > Chapsari (74).

The decrease in RWC in leaves of rice seedlings of almost all varieties was observed. The greatest decrease in RWC was observed in Barakat and Chapsari varieties (by 25 and 26%, respectively). The degree of RWC decrease in Madina, Bakanas, Barakat, and Chapsari can be presented in the following order (% to control, accordingly): Fe norm + Cd (92, 90, 84, and 84) > Fe deficiency − Cd (93, 92, 86, and 83) > Fe deficiency + Cd (82, 79, 75, and 74).

In all the studied varieties, the greatest decrease in RWC was observed in variant “Fe deficiency +Cd” by 18, 21, 25, and 26% in varieties Madina, Bakanas, Barakat, and Chapsari, respectively. The greatest decrease in this variant was found for Barakat and Chapsari varieties.

In all the studied varieties, the greatest decrease in RWC was observed in variant “Fe deficiency+Cd” by 18, 21, 25, and 26% in Madina, Barakat, Bakanas, and Chapsari varieties, respectively. The greatest decrease in this variant was found in the Chapsari variety.

The article "Rice Plants (Oryza sativa L.) under Cd Stress in Fe Deficiency Conditions" was published in 2022. Journal: Biomed Res Int.

The relative water content in Madina, Bakanas, Barakat, and Chapsari varieties was decreased in studied variants in the following order (% to control): Fe deficiency‐Cd (92, 92, 86, and 83) ≥ Fe norm + Cd (91, 90, 84, and 86) > Fe deficiency + Cd (82, 79, 75, and 74). According to obtained results, Cd and Fe deficiency caused a decrease in RWC and the level of decrease under Cd stress in Fe deficiency conditions was the greatest.

According to other research, heavy metals, including Cd, reduce the water content in the plant cell. In conditions of high concentration of heavy metals in growth medium, plants are subjected to osmotic stress, since the osmotic potential of the growing medium will be lower than that in plant cells, so that water is not absorbed by the plant roots [142]. And as a consequence, Cd stress caused a decrease in the stomatal aperture area per unit leaf area [143] and stomatal closing [144]. It was found that the reason for the decrease in the aperture of stomata in *Setaria viridis* plants under Cd stress was the release of potassium and calcium from the stomatal guard cells due to an increase in the permeability of cell membranes [145]. It was also proposed that Cd^2+^ causes stomata closing independently from ABA by entering the cytosol using Ca^2+^ channels [124]. It is supposed that heavy metals slow down the transport of water over short distances in both symplast and apoplast. This decreases the influx of water into the vascular system and affects the supply of water to the aboveground organs.

Water transport over long distances is limited because of a decrease in hydroconductivity in the root, stem, and middle part of the leaf, due to a decrease in the size of conducting vessels, as well as partial lock of xylem vessels by cell debris or gum [124].

There are the opposite data concerning water status of plants under Fe deficiency conditions. It was shown that Fe deficiency causes a decrease in stomatal conductance. It was supposed that Fe deficiency leads to retaining water status in plants [146]. According to other research, levels of stomatal conductivity were close to control or increased, which leads to a loss of stomatal control and causes a decrease in water content in leaves [147].

In our studies, with relative tolerance to Cd and Fe deficiency stresses in Madina and Bakanas varieties, RWC decreased to a lesser extent compared to that in Barakat and Chapsari varieties in all variants. The double stress of Cd and Fe deficiency aggravated their separate negative effect on RWC in leaves of rice plants.

### 3.5. The Effect of Cd and Fe Deficiency on the Proline Content in the Leaves of Rice Seedlings

Proline as an amino acid plays an important role as an osmolite under adverse environmental conditions. Proline was synthesized in tissues capable of rapid cell division, such as shoot apical meristems, in pollen and seeds, where it protects cells from dehydration of cell structures [148].

The article "Rice Plants (Oryza sativa L.) under Cd Stress in Fe Deficiency Conditions" was published in 2022. Journal: Biomed Res Int.

In rice seedlings, the following pattern was observed in proline content (% to control) (Figure 9): Madina variety— Fe deficiency + Cd (206) > Fe norm + Cd (176) = Fe deficiency‐Cd (176); Bakanas variety— Fe deficiency + Cd (133) > Fe deficiency‐Cd (131) > Fe + Cd norm (120); Barakat variety— Fe deficiency + Cd (141) > Fe norm + Cd (133) > Fe deficiency‐Cd (122); and Chapsari variety— Fe deficiency + Cd (128) > Fe norm + Cd (119) > Fe deficiency‐Cd (113).

The level of increase in proline content in different variants among rice varieties can be presented in the following order (% to control): Fe norm+Cd— Madina (178) > Bakanas (120) > Barakat (133) > Chapsari (119); Fe deficiency— Madina (176) > Bakanas (132) > Barakat (122) > Chapsari (113); and Fe deficiency+Cd—Madina (203) > Barakat (141) > Bakanas (133) > Chapsari (128).

In all the studied varieties, the greatest increase in proline content was found in variant “Fe deficiency+Cd” by 103, 33, 41, and 28% in varieties Madina, Bakanas, Barakat, and Chapsari, respectively. In the studied varieties, the proline content increased most in the “Fe deficiency+Cd” variant. Among the varieties, the highest increase in proline was observed in resistant varieties Madina and Bakanas.

Other studies have also observed an increase in proline content in plants exposed to Cd. Proline provides membrane and protein protection at extreme temperatures and excess inorganic ions in the growing medium. Under conditions of osmotic stress, proline is important for the cell, stabilizes proteins, membranes, and subcellular structures, and protects the cell from oxidative stress. The overproduction of proline synthesis led to an increase in the resistance of transgenic tobacco plants to osmotic stress [149, 150]. Proline provides membrane and protein protection under extreme temperatures and excess of inorganic ions [150]. Various transgenes designed to overproduce proline have demonstrated resistance to abiotic stress [151]. A correlative link was found between high levels of proline and the effect of stress factors on plants [149]. Expression of proline in transgenic plants produced increased root biomass under water stress [151]. In transgenic *Arabidopsis* plants, with suppressed proline synthesis, morphological changes, and hypersensitivity to water deficiency, low activity of antioxidant enzymes was found [152]. Under conditions of heavy metal contamination, the synthesis of osmolytes such as proline is one of the ways by which plants fight stress [153, 154]. It is assumed that the accumulation of proline can contribute to osmotic regulation and stabilization of macromolecule structure [155]. Proline also acts as a major source of energy and nitrogen, which can be used to renew growth after stress [156].

The article "Rice Plants (Oryza sativa L.) under Cd Stress in Fe Deficiency Conditions" was published in 2022. Journal: Biomed Res Int.

According to other researchers, under Cd stress (500 *μ*M), the studied rice varieties showed a high content of proline compared to control and the protective effect of proline under osmotic stress was established [157]. It was shown that overexpressing osmolite biosynthesis exhibits increased stress resistance [158]. Fe deficiency, salinity, and the combined effect of these two stresses also caused an increase in the proline content in barley varieties. More resistant to Fe deficiency, varieties showed a higher content of proline in the leaves [150, 159].

### 3.6. Cadmium Effect at Different Fe Status on the Anatomical Structure of the Aboveground Organs of Rice Seedlings

The anatomical structure of leaves and roots under Cd stress in Fe deficiency conditions was studied. In variants with separate effect of Cd and Fe deficiency and joint effect of these stresses, the thickness of the lower epidermis decreased in all varieties (Figures 10 and 11). The lowest decrease was observed in the variant with Fe deficiency. The greatest decrease was observed in the Chapsari variety (by 30, 30, and 50%, accordingly). This parameter decreased in less extent in Madina and Bakanas cvs in all variants. The most decrease in the lower epidermis was observed under double stress of Cd and Fe deficiency.

The thickness of the upper epidermis was also decreased in all variants, but it can be noted that in variant with Fe deficiency, this parameter was decreased in a lesser extent: by 2, 6, 8, and 24% in Madina, Bakanas, Barakat, and Chapsari, respectively (Figures 10 and 12). The thickness of the upper epidermis decreased mostly under joint effect of Cd and Fe deficiency as well as the thickness of the lower epidermis. The Chapsari variety had the greatest decrease (by 52, 34, and 60% under Cd stress and Fe deficiency conditions and under their joint effect, accordingly) in the upper epidermis of leaves in all variants.

The diameter of the conducting bundles of rice varieties of leaves decreased in all studied variants in different degrees (Figures 10 and 13). The greatest changes are observed in the variant “Fe deficiency+Cd.” The smallest changes in the size of the conducting bundles were observed in the variant “Fe norm+Cd.”

Under Fe deficiency stress, the diameter of the conducting bundles decreased in less extent; moreover, in Madina cv, this parameter was on the control level. The greatest changes were also found in the Chapsari variety. Thus, in Fe-deficient conditions, leaf structure changed in less extent. According to other researchers, the Cd effect rather than Fe deficiency alters the leaf anatomy [160, 161]. It was shown that Cd stress and joint effect of Cd and Fe deficiency cause the significant alterations in the leaf anatomy. It was found that under Cd stress, there were changes in the thickness and density of the stomata of the leaves, which can promote an increase in the resistance of the leaves to the metal toxicity [162]. There was a decrease in the thickness of the upper epidermis while the number of stomata and the thickness of the palisade parenchyma increased with Cd toxicity. A decrease in the thickness of the upper epidermis was observed, but at the same time, the number of stomata and the thickness of the palisade parenchyma increased with Cd toxicity. It was observed that the upper epidermis thickness decreased, but at the same time, the thickness of the palisade parenchyma and the number of stomata increased under Cd stress [163].

The article "Rice Plants (Oryza sativa L.) under Cd Stress in Fe Deficiency Conditions" was published in 2022. Journal: Biomed Res Int.

According to the authors, it was observed that the thickness of the abaxial and adaxial sclerenchyma and pericycle was greater under heavy metal (Cu, Cd, Zn, and Pb) stress, and there was a thickening of the epidermis on the abaxial and adaxial sides of the leaves of *Brachiaria decumbens*. It was supposed that it is a strategy for reducing water losses during transpiration, also associated with a large turgor of the leaf blade, which was observed in plants that were contaminated with heavy metals [161]. Some authors have shown an increase in the epidermis thickness and the density of stomata in peanut leaves under Cd stress [164]. In some plant species, depending on their anatomical plasticity, modified leaf tissues appear, which provides better adaptation under stress [165]. It is also known that the number of conducting elements is reduced, an adaptive reaction to ensure the flow of water [166].

### 3.7. Cadmium Effect at Different Fe Status on the Anatomical Structure of the Rice Roots

Anatomical parameters of rice roots changed under Cd and double stress (Fe deficiency+Cd), but differences were not significant. According to the change in the root exodermis, in the variant “Fe norm+Cd,” rice varieties can be arranged in the following order (% to control) (Figures 14 and 15): Madina (110) > Bakanas (97) > Barakat (76) > Chapsari (50). In the presence of Cd, the thickness of the root exodermis in the Chapsari variety decreased to the greatest extent.

At Fe deficiency conditions, a decrease in the thickness of the root exodermis was observed in all the studied rice varieties. In the variant “Fe deficiency-Cd,” the rice varieties by the decrease in this parameter can be presented in the following order: Madina (92) > Bakanas (89) > Barakat (74) > Chapsari (68).

The article "Rice Plants (Oryza sativa L.) under Cd Stress in Fe Deficiency Conditions" was published in 2022. Journal: Biomed Res Int.

In the variant “Fe deficiency+Cd” only in the Madina variety, there was a slight increase (by 7%) in the thickness of the root exodermis; this indicator decreased by 16%, 33%, and 50% in the varieties Bakanas, Barakat, and Chapsari, respectively (% to control): Madina (107) > Bakanas (84) > Barakat (67) > Chapsari (50).

The study of the endodermis thickness under Cd stress and Fe deficiency conditions showed that under Cd stress in varieties Madina and Bakanas, it was slightly increased (by 6% in Madina cv) or stayed on the control level (by 1% in Bakanas cv); in Chapsari and Barakat cvs, this parameter decreased by 21 and 27%, respectively (Figures 14 and 16).

In the variant “Fe norm+Cd,” the endodermis thickness of the varieties can be arranged in the following order (% to control): Madina (106) > Bakanas (101) > Chapsari (79) > Barakat (73).

In the variant “Fe deficiency-Cd,” the thickness of the endodermis decreased in the following order (% to control): Bakanas (100) > Madina (93) > Barakat (84) > Chapsari (79) (Figures 14 and 17). Under Fe deficiency conditions, thickness of the endodermis was on the control level, and in Madina, Barakat, and Chapsari, it decreased by 7, 16, and 21%, accordingly.

Under double stress in the Madina variety, the endodermis thickness decreased in less extent; this parameter decreased by 12, 26, and 36% in Bakanas, Barakat, and Chapsari cvs, respectively.

In the variant “Fe deficiency+Cd,” the thickness of the endodermis decreased in all the studied rice varieties (in % to control): Madina (96) > Bakanas (88) > Barakat (74) > Chapsari (64).

The diameter of the central cylinder of roots in the tolerant variety Madina slightly increased under Cd stress. In other varieties which decreased in different levels, the most decrease was observed in Chapsari cv.

According to the change in the diameter of the central cylinder in the “Fe norm+Cd” variant, the varieties are arranged as follows (% to control) (Figures 14and 16): Madina (107) > Bakanas (96) > Barakat (91) > Chapsari (64).

The varieties in the variant “Fe deficiency-Cd” by the change of this indicator are arranged as follows (% to control): Madina (99) ≥ Bakanas (98) > Barakat (88) > Chapsari (67). Under Fe deficiency stress, the Chapsari variety was distinguished by the most decrease in the diameter of the central cylinder.

Under double stress, the same pattern has been preserved.

The article "Rice Plants (Oryza sativa L.) under Cd Stress in Fe Deficiency Conditions" was published in 2022. Journal: Biomed Res Int.

In the variant “Fe deficiency+Cd,” varieties can be arranged in the following order (in % to control): Bakanas (99) > Madina (94) > Barakat (81) > Chapsari (55).

In resistant Madina cv, the exodermis of roots slightly increased under Cd and double stress (Fe deficiency+Cd) (by 10 and 7%, respectively), as well as endodermis thickness and the diameter of the central cylinder under Cd stress (by 6 and 7%); in other varieties, all root anatomical parameters do not change or have tendency to decrease, but the differences were not significant. The alterations in anatomical structure of plant roots were observed by other researchers. According to other studies, the diameter of the roots of *Cicer arietinum* L. decreased under Cd stress. The endodermal cells of the Cd-treated roots had smaller size and thick walls than those of the control plant roots. The stem diameter decreased due to the reduction in the size of cells and vascular elements under Cd stress [167]. In chickpea plants, the area of cortical stem cells was smaller due to the action of Cd compared to control plants.

Xylem vessels in Cd-treated plants had smaller size, and their number also decreased. The area of vessels in the treated Cd leaves became smaller compared to that in the control leaves.

A decrease in the thickness of the leaves and in the area of the vessels and the closure of the stomata compared to the control sample were observed [168]. Other researchers have shown that the thickness of the exodermis and endodermis of roots, xylem cell walls, and cortical parenchyma in *Brachiaria decumbens* thickens with increasing heavy metal content in the growing medium [161]. The thickness of the exodermis and endoderm of plants roots increased under the conditions of contamination. It is assumed that the destruction of the epidermal tissue was compensated by the thickening of the exodermis tissue [169]. The endodermis and exodermis of plant roots are of great importance in protecting plants from various stress factors [170]. During the study of the heavy metals' effect on the plant *Brachiaria decumbens*, it is assumed that the thickening of the root exodermis and endodermis is a response to reduce the metal translocation from roots to shoots. This property indicates a high tolerance to heavy metals and may be a plant strategy to minimize the transfer of metals to aboveground organs. An increase in the thickness of the exodermis and endodermis in roots of plants indicates a high resistance to heavy metals [169]. The thickening of the exodermis and endodermis indicates a better ability to prevent the apoplastic movement of the metal, and the increase in cell wall thickness contributes to the accumulation of heavy metals in the roots, reducing their movement to aboveground organs. Caspari belts reduce the surface of the membrane available for ion absorption [171]. The lowering of the epidermal layer of leaves was observed by other authors. The decrease in the thickness of plant leaves observed by other researchers is explained by the flattening of epidermal cells, which results in a reduction in intercellular spaces in mesophyll tissues [172].

The article "Rice Plants (Oryza sativa L.) under Cd Stress in Fe Deficiency Conditions" was published in 2022. Journal: Biomed Res Int.

## 4. Conclusion

Cadmium contamination of the soil due to the functioning of metallurgical plants and the widespread use of phosphorus fertilizers aggravated by the unbalanced mineral composition of the soil is a big problem in developing countries. The importance of this work is that a comprehensive study at the physiological, biochemical, and anatomical level of Cd effect under Fe deficiency conditions on various rice varieties was carried out. The degree of reduction of all studied parameters under double stress was the greatest compared to other variants, which indicates that a decrease in the Fe content in the nutrient medium exacerbates the toxic effect of Cd. This indicates the need for a full-fledged plant mineral nutrition, especially Fe, under Cd stress. Based on obtaining integral indicators under the joint effect of Cd and Fe deficiency conditions, it can be concluded that plant responses at the physiological, biochemical, and anatomical levels in resistant rice varieties were expressed to a greater extent compared to those in Cd-sensitive varieties. The identification of relatively resistant and sensitive varieties to the effects of double stress and revealed variety specificity of rice plant responses allow assuming differences in plant response mechanisms against the joint effect of Cd and deficiency of Fe, also in the activity of genes, responsible for the transport of these metals in rice varieties. The further investigation of the influence of Fe-containing fertilizers on these rice varieties to decrease the toxicity of Cd, in order to reveal the mechanisms of their effect at the physiological and biochemical level, as well as the study of Fe and Cd transporter genes at the molecular level, is needed. The further study of the expression of Cd and Fe transporter genes will expand knowledge about the genetic determinacy of plant responses to stress and use them to reduce the unfavorable impact of Fe deficiency for plants.

## Figures and Tables

**Figure 1:** The effect of Cd and Fe deficiency on the biomass accumulation in aboveground organs of 14 d rice seedlings. Control-Fe norm-Cd: nutrient medium (NM)+100 *μ*М Fe; Fe norm+Cd: NM+100 *μ*М Fe+200 *μ*М Сd; Fe deficiency-Cd: NM+0 *μ*М Fe; Fe deficiency+Cd: NM+0 *μ*М Fe+200 *μ*М Сd. Vertical bars represent ±SE of three replicates (*n* = 3); the differences within variety between control and treatments: ^∗^*p* < 0.1, ^∗∗^*p* < 0.05, and ^∗∗∗^*p* < 0.01; the differences across varieties are significant at *p* < 0.001.

The article "Rice Plants (Oryza sativa L.) under Cd Stress in Fe Deficiency Conditions" was published in 2022. Journal: Biomed Res Int.

**Figure 2:** The effect of Cd and Fe deficiency on the length of aboveground organs of 14 d rice seedlings. Control-Fe norm-Cd: nutrient medium (NM)+100 *μ*М Fe; Fe norm+Cd: NM+100 *μ*М Fe+200 *μ*М Сd; Fe deficiency-Cd: NM+0 *μ*М Fe; Fe deficiency+Cd: NM+0 *μ*М Fe+200 *μ*М Сd. Vertical bars represent ±SE of three replicates (*n* = 3); the differences within variety between control and treatments: ^∗^*p* < 0.1; ^∗∗^*p* < 0.05, and ^∗∗∗^*p* < 0.01; the differences across varieties are significant at *p* < 0.001

**Figure 3:** The effect of Cd and Fe deficiency on root biomass of 14 d rice seedlings. Control-Fe norm-Cd: nutrient medium (NM)+100 *μ*М Fe; Fe norm+Cd: NM+100 *μ*М Fe+200 *μ*М Сd; Fe deficiency-Cd: NM+0 *μ*М Fe; Fe deficiency+Cd: NM+0 *μ*М Fe+200 *μ*М Сd. Vertical bars represent ±SE of three replicates (*n* = 3); the differences within variety between control and treatments: ^∗^*p* < 0.1, ^∗∗^*p* < 0.05, and ^∗∗∗^*p* < 0.01; the differences across varieties are significant at *p* < 0.001.

**Figure 4:** The effect of Cd and Fe deficiency on the root length of 14 d rice seedlings. Control-Fe norm-Cd: nutrient medium (NM)+100 *μ*М Fe; Fe norm+Cd: NM+100 *μ*М Fe+200 *μ*М Сd; Fe deficiency-Cd: NM+0 *μ*М Fe; Fe deficiency+Cd: NM+0 *μ*М Fe+200 *μ*М Сd. Vertical bars represent ±SE of three replicates (*n* = 3); the differences within variety between control and treatments: ^∗^*p* < 0.1, ^∗∗^*p* < 0.05, and ^∗∗∗^*p* < 0.01; the differences across varieties are not significant at *p* > 0.05.

**Figure 5:** The effect of Cd and Fe deficiency on the content of chlorophyll *a* in the leaves of 14 d rice seedlings. Сontrol-Fe norm-Cd: nutrient medium (NM)+100 *μ*М Fe; Fe norm+Cd: NM+100 *μ*М Fe+200 *μ*М Сd; Fe deficiency-Cd: NM+0 *μ*М Fe; Fe deficiency+Cd: NM+0 *μ*М Fe+200 *μ*М Сd. Vertical bars represent ±SE of three replicates (*n* = 3); the differences within variety between control and treatments: ^∗^*p* < 0.1, ^∗∗^*p* < 0.05, and ^∗∗∗^*p* < 0.01; the differences across varieties are significant at *p* < 0.001.

**Figure 6:** Effect of Cd and Fe deficiency on the content of chlorophyll *b* in the leaves of 14 d rice seedlings. Сontrol-Fe norm-Cd: nutrient medium (NM)+100 *μ*М Fe; Fe norm+Cd: NM+100 *μ*М Fe+200 *μ*М Сd; Fe deficiency-Cd: NM+0 *μ*М Fe; Fe deficiency+Cd: NM+0 *μ*М Fe+200 *μ*М Сd. Vertical bars represent ±SE of three replicates (*n* = 3); the differences within variety between control and treatments: ^∗^*p* < 0.1, ^∗∗^*p* < 0.05, and ^∗∗∗^*p* < 0.01; the differences across varieties are significant at *p* < 0.001.

The article "Rice Plants (Oryza sativa L.) under Cd Stress in Fe Deficiency Conditions" was published in 2022. Journal: Biomed Res Int.

**Figure 7:** The effect of Cd and Fe deficiency on the content of carotenoids in the leaves of 14 d rice seedlings. Сontrol-Fe norm-Cd: nutrient medium (NM)+100 *μ*М Fe; Fe norm+Cd: NM+100 *μ*М Fe+200 *μ*М Сd; Fe deficiency-Cd: NM+0 *μ*М Fe; Fe deficiency+Cd: NM+0 *μ*М Fe+200 *μ*М Сd. Vertical bars represent ±SE of three replicates (*n* = 3); the differences within variety between control and treatments: ^∗^*p* < 0.1, ^∗∗^*p* < 0.05, and ^∗∗∗^*p* < 0.01; the differences across varieties are not significant (*p* > 0.05).

**Figure 8:** The effect of Cd and Fe deficiency on the relative water content (RWC) in the leaves of 14 d rice seedlings. Сontrol-Fe norm-Cd: nutrient medium (NM)+100 *μ*М Fe; Fe norm+Cd: NM+100 *μ*М Fe+200 *μ*М Сd; Fe deficiency-Cd: NM+0 *μ*М Fe; Fe deficiency+Cd: NM+0 *μ*М Fe+200 *μ*М Сd. Vertical bars represent ±SE of three replicates (*n* = 3); the differences within variety between control and treatments: ^∗^*p* < 0.1, ^∗∗^*p* < 0.05, and ^∗∗∗^*p* < 0.01; the differences across varieties are significant (*p* < 0.001).

**Figure 9:** The effect of Cd and Fe deficiency on proline content in the leaves of 14 d rice seedlings. Сontrol-Fe norm-Cd: nutrient medium (NM)+100 *μ*М Fe; Fe norm+Cd: NM+100 *μ*М Fe+200 *μ*М Сd; Fe deficiency-Cd: NM+0 *μ*М Fe; Fe deficiency+Cd: NM+0 *μ*М Fe+200 *μ*М Сd. Vertical bars represent ±SE of three replicates (*n* = 3); the differences within variety between control and treatments: ^∗^*p* < 0.1, ^∗∗^*p* < 0.05, and ^∗∗∗^*p* < 0.01; the differences across varieties (*p* < 0.05) are significant

**Figure 10:** Anatomical structures of 14 d rice seedling leaves: (A) control-Fe norm-Cd—nutrient medium (NM)+100 *μ*М Fe, (B) Fe norm+Cd—NM+100 *μ*М Fe+200 *μ*М Сd, (C) Fe deficiency-Cd—NM+0 *μ*М Fe, and (D) Fe deficiency+Cd—NM+0 *μ*М Fe+200 *μ*М Сd. 1—lower epidermis, 2—upper epidermis, and 3—conducting bundles.

**Figure 11:** Effect of Cd under different Fe status on the thickness of the lower epidermis of 14 d rice seedlings. Control-Fe norm-Cd: nutrient medium (NM)+100 *μ*М Fe; Fe norm+Cd: NM+100 *μ*М Fe+200 *μ*М Сd; Fe deficiency-Cd: NM+0 *μ*М Fe; Fe deficiency+Cd: NM+0 *μ*М Fe+200 *μ*М Сd. Vertical bars represent ±SE of three replicates (*n* = 3); the differences within variety between control and treatments: ^∗^*p* > 0.05, ^∗∗^*p* < 0.05, and ^∗∗∗^*p* < 0.01; the differences across varieties (*p* < 0.001) are significant.

**Figure 12:** Effect of Cd under different Fe status on the thickness of the upper epidermis of leaves of rice seedlings. Control-Fe norm-Cd: nutrient medium (NM)+100 *μ*М Fe; Fe norm+Cd: NM+100 *μ*М Fe+200 *μ*М Сd; Fe deficiency-Cd: NM+0 *μ*М Fe; Fe deficiency+Cd: NM+0 *μ*М Fe+200 *μ*М Сd. Vertical bars represent ±SE of three replicates (*n* = 3); the differences within variety between control and treatments: ^∗^*p* > 0.05, ^∗∗^*p* < 0.05, and ^∗∗∗^*p* < 0.01; the differences across varieties (*p* < 0.001) are significant.

The article "Rice Plants (Oryza sativa L.) under Cd Stress in Fe Deficiency Conditions" was published in 2022. Journal: Biomed Res Int.

**Figure 13:** Effect of Cd under different Fe status on the diameter of conducting bundles of leaf rice seedlings. Control-Fe norm-Cd: nutrient medium (NM)+100 *μ*М Fe; Fe norm+Cd: NM+100 *μ*М Fe+200 *μ*М Сd; Fe deficiency-Cd: NM+0 *μ*М Fe; Fe deficiency+Cd: NM+0 *μ*М Fe+200 *μ*М Сd. Vertical bars represent ±SE of three replicates (*n* = 3); the differences within variety across treatments: ^∗^*p* > 0.05, ^∗∗^*p* < 0.05, and ^∗∗∗^*p* < 0.01; the differences across varieties (*p* < 0.001) are significant.

**Figure 14:** Anatomical structures of 14 d rice seedling leaves: (A) control-Fe norm-Cd—nutrient medium (NM)+100 *μ*М Fe, (B) Fe norm+Cd—NM+100 *μ*М Fe+200 *μ*М Сd, (C) Fe deficiency-Cd—NM+0 *μ*М Fe, and (D) Fe deficiency+Cd—NM+0 *μ*М Fe+200 *μ*М Сd. 1—exodermis, 2—endodermis, and 3—central cylinder.

**Figure 15:** Effect of Cd under different Fe status on the thickness of the exodermis of roots of rice seedlings. Control-Fe norm-Cd: nutrient medium (NM)+100 *μ*М Fe; Fe norm+Cd: NM+100 *μ*М Fe+200 *μ*М Сd; Fe deficiency-Cd: NM+0 *μ*М Fe; Fe deficiency+Cd: NM+0 *μ*М Fe+200 *μ*М Сd. Vertical bars represent ±SE of three replicates (*n* = 3); the differences within variety between control and treatments: ^∗^*p* > 0.05, ^∗∗^*p* < 0.05, and ^∗∗∗^*p* < 0.01; the differences across varieties (*p* < 0.001) are significant.

**Figure 16:** Effect of Cd under different Fe status on the diameter of the central cylinder of roots of rice seedlings. Control-Fe norm-Cd: nutrient medium (NM)+100 *μ*М Fe; Fe norm+Cd: NM+100 *μ*М Fe+200 *μ*М Сd; Fe deficiency-Cd: NM+0 *μ*М Fe; Fe deficiency+Cd: NM+0 *μ*М Fe+200 *μ*М Сd. Vertical bars represent ± SE of three replicates (*n* = 3); the differences within variety between control and treatments: ^∗^*p* > 0.05, ^∗∗^*p* < 0.05, and ^∗∗∗^*p* < 0.01; the differences across varieties (*p* < 0.001) are significant.

**Figure 17:** Effect of Cd under different Fe status on the thickness of the endodermis of roots of rice seedlings. Control-Fe norm-Cd: nutrient medium (NM)+100 *μ*М Fe; Fe norm+Cd: NM+100 *μ*М Fe+200 *μ*М Сd; Fe deficiency-Cd: NM+0 *μ*М Fe; Fe deficiency+Cd: NM+0 *μ*М Fe+200 *μ*М Сd. Vertical bars represent ±SE of three replicates (*n* = 3); the differences within variety between control and treatments: ^∗^*p* > 0.05, ^∗∗^*p* < 0.05, and ^∗∗∗^*p* < 0.01; the differences across varieties (*p* < 0.001) are significant.

The article "Rice Plants (Oryza sativa L.) under Cd Stress in Fe Deficiency Conditions" was published in 2022. Journal: Biomed Res Int.

## Data Availability

We have not put any data concerning our results in any archived datasets.
